The article "Cerebral Microbleed Detection via Convolutional Neural Network and Extreme Learning Machine" was retracted in 2023. Reasons: compromised peer review; unreliable results or conclusions.

# Cerebral Microbleed Detection *via* Convolutional Neural Network and Extreme Learning Machine

**DOI:** 10.3389/fncom.2021.738885

**Published:** 2021-09-10

**Authors:** Siyuan Lu, Shuaiqi Liu, Shui-Hua Wang, Yu-Dong Zhang

**Affiliations:** ^1^School of Informatics, University of Leicester, Leicester, United Kingdom; ^2^College of Electronic and Information Engineering, Hebei University, Baoding, China; ^3^School of Mathematics and Actuarial Science, University of Leicester, Leicester, United Kingdom

**Keywords:** computer-aided diagnosis, deep learning, convolutional neural network, extreme learning machine, bat algorithm

## Abstract

**Aim:** Cerebral microbleeds (CMBs) are small round dots distributed over the brain which contribute to stroke, dementia, and death. The early diagnosis is significant for the treatment.

**Method:** In this paper, a new CMB detection approach was put forward for brain magnetic resonance images. We leveraged a sliding window to obtain training and testing samples from input brain images. Then, a 13-layer convolutional neural network (CNN) was designed and trained. Finally, we proposed to utilize an extreme learning machine (ELM) to substitute the last several layers in the CNN for detection. We carried out an experiment to decide the optimal number of layers to be substituted. The parameters in ELM were optimized by a heuristic algorithm named bat algorithm. The evaluation of our approach was based on hold-out validation, and the final predictions were generated by averaging the performance of five runs.

**Results:** Through the experiments, we found replacing the last five layers with ELM can get the optimal results.

**Conclusion:** We offered a comparison with state-of-the-art algorithms, and it can be revealed that our method was accurate in CMB detection.

## Introduction

Cerebral microbleeds (CMBs) are caused by cerebral small vessel diseases, which often occur among the elderly. CMBs are also related to age, blood pressure, and cardiopathy. CMBs can contribute to stroke, cognition impairment, dementia, and even death. CMBs appear as tiny round dots distributed over the brain on T2 weighted magnetic resonance images. The accurate detection of CMBs at its early stage poses a challenge because it is tedious and difficult to find CMBs with naked eyes. Therefore, developing an automatic CMB detection system is significant and necessary. Benefited from the rapid advancement of deep learning and pattern recognition, over the last decade, researchers have proposed many CMB detection methods.

Barnes et al. (2011) put forward a semi-automated detection method for CMB. They firstly leveraged a threshold algorithm to obtain hypointensities in brain MRI. Then, they proposed to use a support vector machine (SVM) to identify CMB and the hypointensities. Finally, the result was refined by manual intervention. The proposed method sacrificed some detection sensitivity for less detection time. Kuijf et al. (2012) used radial symmetry transform to get potential CMBs from both echoes of magnetic resonance sequence. Two raters were responsible for checking the result. Bian et al. (2013) employed 2D fast radial symmetry transform (RST) to generate potential CMB regions. Afterward, a 3D region growing method was performed on the candidate regions, and geometric features were used to eliminate false candidates. Fazlollahi et al. (2015) suggested leveraging multi-scale Laplacian of Gaussian algorithm to get possible CMB with their background. Then, 3D shape features were calculated from the possible CMBs. Finally, a cascade of binary random forests was trained to identify those candidates as CMB or non-CMB. Ourselin et al. (2015) proposed to utilize multiple radial-symmetry transforms to detect spherical structures from susceptibility-weighted images (SWI) and used the patches to form feature vectors. A random forest was trained for segmentation. Kaaouana et al. (2016) used internal field maps to rate the CMBs from susceptibility-weighted images. Zhang et al. (2017a) introduced artificial neural networks to CMB detection. They generated the experimental dataset by slicing neighborhood processing. A 3-layer neural network was trained using early stopping for classification. In their experiment, they compared several activation functions, including the leaky rectified linear unit, rectified linear unit, and logistic sigmoid, and found out the performance of the leaky rectified linear unit was better. Later, Zhang et al. (2017b) constructed a 7-layer deep neural network to detect CMB, and the classification accuracy was further improved. Chen et al. (2018) suggested employing a 3D deep residual network for CMB diagnosis. The residual blocks include convolution and batch normalization. Hong (2018a) built a convolutional neural network (CNN) for CMB detection. They tested all the hyper-parameters to improve the classification performance. Hong (2019) employed ResNet to extract features and introduced transfer learning to detect CMBs. Their system yielded good classification performance in the experiment. Liu et al. (2020) proposed to fuse the information in the space domain as well as the Fourier domain to generate the CMB candidates. Chesebro et al. (2021) used a 2D gradient map and the circular Hough transform to obtain the initial CMBs and removed the false positive ones by entropy and blob analysis.

The article "Cerebral Microbleed Detection via Convolutional Neural Network and Extreme Learning Machine" was retracted in 2023. Reasons: compromised peer review; unreliable results or conclusions.

From the above literature, we can find that a computer-aided diagnosis system based on medical images usually consists of these modules: image pre-processing, feature extraction, classifier training, and testing. For CMB detection, researchers often segment the images to generate potential CMBs and then eliminate the false ones. However, image segmentation can be time-consuming and suffer from low accuracy. The distribution of image features is also significant because it decides the complexity of the classification problem. Hand-crafted features may be domain-dependent, which means the features are effective only in certain datasets but cannot be transferred to all the datasets. One of the problems in classifier training is overfitting, where the trained classifier works accurately on the training set but poorly on the testing set. Overfitting tends to occur on small datasets and deep learning models which contain too many parameters.

In this study, a novel CMB detection approach was proposed, which combined CNN and extreme learning machine (ELM). CNN was trained for automatic feature extraction, and ELM was trained for final classification. To obtain better classification performance, the parameters in ELM were further optimized by bat algorithm (BA), which belongs to a swarm intelligence method. We combined CNN and ELM-BA by substituting the last *n* layers of the deep convolutional network by ELM-BA. We proposed a searching algorithm to determine the best value of *n*. The classification performance of our method was obtained by 5 × hold-out validation (HV). In the experiment on a CMB dataset containing over 10,000 samples, the proposed system achieved good classification performance compared to the state of the arts.

The rest of this paper is organized as following sections: Section 2 presents the CMB dataset in our experiment, the methods are given in Section 3, Section 4 is about hyper-parameter settings and platform of the experiment, the results’ comparison is provided in Section 5, and Section 6 offers our conclusion.

## Materials

### Data Description

The dataset in our evaluation experiments is the same as the one used in the previous work (Zhang et al., 2017b). The volume of the 3D images is 364 × 448 × 48, reconstructed by Syngo MR B17 software. The images are labeled in voxel-level by three experienced radiologists under the guidance of the microbleed anatomical rating scale (MARS). The vessels and the large lesions (over 10mm) were excluded. All the possible and definite voxels are regarded as CMBs in this paper.

### Sliding Neighborhood Processing

To generate the dataset for classifier training and testing, sliding neighborhood processing (SNP) was employed. SNP works with a window sliding over the SWIs to generate smaller images as the samples (shown in Figure 1). As for the labels, the sample will be labeled as CMB if the center pixel is in a CMB. Otherwise, it will be labeled as non-CMB. Some generated samples are listed in Figure 2.

The article "Cerebral Microbleed Detection via Convolutional Neural Network and Extreme Learning Machine" was retracted in 2023. Reasons: compromised peer review; unreliable results or conclusions.

**FIGURE 1:** Diagram of SNP.

**FIGURE 2:** Samples in our dataset.

## Methods

Conventionally, image-based computer-aided diagnosis systems firstly generate features from the input image. Then, those features were used to train a classification model. Traditional algorithms employ various hand-crafted features to form the feature vector (Pan et al., 2014; Chen and Chen, 2016; Zhan and Chen, 2016; Liu, 2017; Wang et al., 2018), but hand-crafted features are usually domain-dependent and fail in scalability. Moreover, useful classification information can be lost during hand-crafted feature extraction. So, we leverage CNN for feature extraction. Using convolution layers and pooling layers, CNN can generate features from simple representation to complex representation automatically (Li et al., 2017; Nogueira et al., 2017; Sun et al., 2017). However, the fully connected layers located at the end of the CNN can result in overfitting with backpropagation algorithms. ELM belongs to training methods for networks with three layers. The training of ELM is over one thousand times faster than traditional algorithms, but its generalization performance is good (Guang-Bin et al., 2006; Huang et al., 2006a). Therefore, we replaced the fully connected layers with ELM and optimized the parameters in ELM using the bat algorithm (BA) to further boost its classification performance.

### Convolutional Neural Network

Convolutional neural network is not a new structure in artificial intelligence. It was developed by Yann LeCun as early as 1989, but restricted by the hardware and the lack of efficient training algorithm, CNN was not widely applied at that time. CNN became a dominant architecture in image processing and recognition after the amazing classification performance was achieved on the ImageNet (Krizhevsky et al., 2012). After that, every year there are new CNNs invented, such as VGG (Simonyan and Zisserman, 2015), ResNet (He et al., 2016), DenseNet (Huang et al., 2016), etc., which kept breaking the record of the competition.

Basically, a CNN includes three different types of layers (Hong et al., 2019; Yu and Wang, 2019). The convolution layer serves as a feature extractor, the pooling layer is used to reduce the dimension of features, and the fully connected layer is often arranged at the end of the CNN for recognition and classification.

The article "Cerebral Microbleed Detection via Convolutional Neural Network and Extreme Learning Machine" was retracted in 2023. Reasons: compromised peer review; unreliable results or conclusions.

The convolution layer employs a set of kernel filters to scan the image and generate feature maps, as is shown in Figure 3. The kernels are assigned with weights to be trained. For feature map *I* in size of (*U,V*) and a kernel *K* in size of (*p*,*q*), the convolution operation expression is


(1) $$C=\left(I*K\right)\,\left(x,y\right)=\sum_{U}\sum_{V}I\,\left(x-p,y-q\right)\times K\,\left(p,q\right)$$

**FIGURE 3:** A simple example of convolution.

The obtained feature maps from early convolution layers are large in volume, so the pooling layer is followed to shrink the feature dimensions. Pooling operation sweeps the feature maps with a window of fixed size and produces the reduced map by some strategies like max, min, and average pooling for different purposes (shown in Figure 4).

**FIGURE 4:** Pooling operations.

A fully connected layer (FCL) is a common network structure (Jiang, 2017; Hong, 2018b; Sui, 2018). Each node in FCLs is connected with each node in its adjacent layers. The links are assigned with weights and biases.

The activation function is another important part of an artificial neural network, which was inspired by the activation in human neurons. In neural networks, the activation function provides non-linearity mapping and complex approximation ability. There are a bunch of activation functions to choose from, like sigmoid function, radial basis function, cosine function, hard limit function, and rectified linear unit (ReLU). ReLU is effective for deep models because it is simple to compute. The expression of ReLU is


(2) $$\text{ReLU}\,\left(x\right)=\max\left(0,x\right)=\left\{ \begin{array}{c} x,x\geq 0\\ 0,x<0 \end{array}\right.$$

At the last layer of CNN, the softmax function is often employed to convert the output of the fully connected layer into probabilities which can avoid the overflow problem. The formula of softmax is


(3) $$\text{softmax}\,{\left(x\right)}_{i}=\frac{\exp\left(x_{i}\right)}{\sum_{j=1}^{n}\exp\left(x_{j}\right)}$$

With all the above methods, a CNN is built, and its parameters can be trained by stochastic gradient descent with momentum (SGDM).

### Extreme Learning Machine

Convolutional neural network is effective in image recognition, but its performance can be improved by replacing its fully connected layers with other efficient classifiers. In this study, ELM was chosen, which is a novel training approach for SLFN (Li, 2019), shown in Figure 5. Gradient descent algorithms are widely applied in various applications, but they require many iterations to converge, which is computationally expensive. The solutions obtained by gradient descent may be only the local best instead of the global best.

The article "Cerebral Microbleed Detection via Convolutional Neural Network and Extreme Learning Machine" was retracted in 2023. Reasons: compromised peer review; unreliable results or conclusions.

**FIGURE 5:** Structure of ELM.

Extreme Learning Machine trains in a different way, which converges within three steps. Suppose the data for training is


(4) $$M=\left[\left(x_{i},y_{i}\right)|x_{i}\in R^{n},y_{i}\in R^{m},i=1,\ldots ,N\right]$$

Firstly, ***w****_*i*_* and *b*_*i*_ are pre-defined randomly. With the training samples, we can get the activation **H** in the hidden layer. Finally, the output weights β can be determined using the pseudo-inverse.


(5) $$\beta ={\text{H}}^{*}\,Y$$

In which Y = (*y*_1_, *y*_2_,…, *y*_*N*_)^*T*^ and **H^∗^** denotes the pseudo-inverse matrix. (*o*_1_,…, *o*_*m*_) is the output of ELM. The rigorous proof is given in literatures (Li et al., 2005; Guang-Bin et al., 2006; Huang et al., 2006b, 2015). The training steps are summarized in Table 1.

**TABLE 1:** ELM training steps.

Training of ELM
Input: the labeled data for training, see Equation 4.
Step1: Random initialization of weights *w*_*i*_ and biases *b*_*i.*_ in the input layer
Step2: Calculate the hidden layer activation matrix H using the training set.
Step3: Determine the output weights β using Equation 5.
Output: the trained ELM

Extreme learning machine learns much faster than traditional gradient descent methods, and its generalization is good as well. Due to its simple implementation and outstanding performance, ELM is now becoming more and more popular in real applications (Zou et al., 2017; Huang et al., 2018; Liu et al., 2018), and its variants have also emerged (Golestaneh et al., 2018; Yang et al., 2018; Xia, 2019).

### Bat Algorithm

The input parameters in ELM are initialized randomly and stay fixed in the whole learning process, which probably hampers the generalization performance. So, we proposed to leverage a bat algorithm to optimize these parameters to improve the classification performance and robustness.

BA belongs to a swarm optimization method, which was developed by the preying of bats (Yang, 2010). BA employs a set of bats, and each bat contains one potential solution in the solution space of D-dimensions. The bats search the space using ultrasound of different loudness and frequencies, and the fitness values are calculated. Solutions with better fitness values will substitute those with worse fitness values. Given a fitness function of *f*(***x***) to be minimized and target solution


(6) $$x={\left(x_{1},x_{2},\ldots ,x_{d}\right)}^{\text{T}}$$

The steps of BA are offered in Table 2.

**TABLE 2:** Pseudocode of BA optimization.

Input: Fitness function *f*(***x***)
Output: The optimal solution: ***x***^∗^ = (*x*_1_, *x*_2_,…, *x*_*d*_)^*T*^ and its fitness
Randomly initialize a set of bats in the solution space, and define the loudness attenuation factor α, the max pulse loudness A_0_, the max pulse rate R_0_, the frequency enhancement factor γ, the max iteration *i_max*, and the searching frequency range [*f*_*min*_, *f*_*max*_]. While (the max iteration has not been reached) {
Calculate the fitness values of each bat according to their location ***x***_*i*_. Update the searching pulse frequency, velocity, and location of bats by Equations 7–9. Generate a random value *rand* if *rand* > γ_*i*_ A new solution random is generated using Equation 10. if *rand* < A_*i*_ && *f*(***x***_*i*_) > *f*(***x***^∗^) Substitute the best solution with the generated one and update the parameters by Equations 11, 12. Sort the fitness of bats and find out the best solution so far }

Important operations:

• Updating the bats:

(7) $$f_{i}=f_{m\,i\,n}+\left(f_{m\,a\,x}-f_{m\,i\,n}\right)\times \beta$$

(8) $$v_{i}^{t}=v_{i}^{t-1}+\left(x_{i}^{t}-x^{*}\right)\times f_{i}$$

(9) $$x_{i}^{t}=x_{i}^{t-1}+v_{i}^{t}$$

In which *f*_*i*_ denotes the searching frequency of the *i*^*th*^ bat, β is a random variable from [0,1], $v_{i}^{t}$ and $v_{i}^{t-1}$ stand for the velocities of the *i*^*th*^ bat in iteration *t* and *t*-1, $x_{i}^{t}$ and $x_{i}^{t-1}$ denote the potential solutions of the *i*^*th*^ bat in iteration *t* and *t*-1, and ***x***^∗^ denotes the best solution obtained by all the bats at that time.

• Generating a new solution:

(10) $$x_{\mathrm{new}}=x_{\mathrm{old}}+\varepsilon \,A^{t}$$

Where ε denotes a random value from (−1, 1), and *A*^*t*^ denotes the mean value of loudness of all bats at that iteration.

• Updating parameters:

(11) $$A_{i}^{t+1}=\alpha \times A_{i}^{t}$$

(12) $$r_{i}^{t+1}=R_{0}\times \left(1-e^{-\gamma \,t}\right)$$

The diagram of BA is illustrated below in Figure 6.

The article "Cerebral Microbleed Detection via Convolutional Neural Network and Extreme Learning Machine" was retracted in 2023. Reasons: compromised peer review; unreliable results or conclusions.

**FIGURE 6:** BA diagram.

For training ELM, the fitness is the loss function, and the bats are the weights and biases. The mean-squared error (MSE) of the ELM output and the sample label served as the fitness function in our BA optimization:


(13) $$\begin{array}{c} F\,i\,t\,n\,e\,s\,s=M\,S\,E\\ =\sum_{i=1}^{N}{\left(o_{i}-y_{i}\right)}^{2} \end{array}$$

where *o*_*i*_ denotes the ELM output and *y*_*i*_ represents the expected output. In every iteration of BA optimization, the parameters in bats will be reshaped to form weights and biases in the ELMs. The MSE will be calculated using the training set.

### Proposed Method: CNN-ELM-BA

Combining convolutional neural network, extreme learning machine, and bat algorithm, we proposed the CMB detection method abbreviated as CNN-ELM-BA. Firstly, a 13-layer CNN was trained using SGDM, and the detailed information is given in Table 3. The architecture of our CNN was determined with our empirical experience.

**TABLE 3:** Parameters in CNN.

#	Name	Type	Description
1	“input”	Input Image	Images of 41 × 41 × 1
2	“conv1”	Convolution layer	2 3 × 3 × 1 convolutions, stride 1 and padding 2
3	“relu1”	ReLU activation	ReLU activation function
4	“maxpool1”	Max Pooling	2 × 2 max pooling, stride 1 and no padding
5	“conv2”	Convolution layer	2 3 × 3 × 2 convolutions, stride 1 and padding 2
6	“relu2”	ReLU activation	ReLU activation function
7	“maxpool2”	Max Pooling	2 × 2 max pooling, stride 1 and no padding
8	“fc1”	Fully Connected layer	An FCL with 32 nodes
9	“relu3”	ReLU activation	ReLU activation function
10	“dropout”	Dropout layer	50% dropout layer
11	“fc2”	Fully Connected layer	An FCL with 2 nodes
12	“softmax”	Softmax	Softmax mapping
13	“output”	Classification Output layer	Types: “non-CMB” and “CMB”

Then, to boost the classification performance, an ELM was used to replace the last *n* layers of CNN for classification. Finally, the BA was leveraged to train the parameters in the ELM on the training set.

To find the optimal value of *n*, we proposed a searching algorithm. We run our system to get the classification results of our CNN-ELM-BA using a set of n values ranging from 3 to 7, which was correspondent to “fc_2” to “maxpool_2” of CNN. We selected to replace the layers after “maxpool_2” because the convolution and pooling operations are closely related to image representation generation. Moreover, the dimension of output features in early layers is too large for an image of 41 × 41 pixels. The number of the output features in “fc_2” is only 32, which is suitable for classifier training.

The pseudocode and flowchart of CNN-ELM-BA are given below in Table 4 and Figure 7, respectively. The pseudocode of the searching method is presented in Table 5.

**TABLE 4:** Pseudocode of our CNN-ELM-BA (run five times).

Input: The labeled training and testing set.
Step1: Train the 13-layer CNN using training set by SGDM with hyperparameters: MiniBatchSize = 60, MaxEpochs = 10, InitialLearnRate = 1e-2.
Step2: Use an ELM structure to substitute the last *n* layers of the CNN.
Step3: Optimize the weights and biases in the ELM using the bat algorithm.
Step4: Evaluate the generalization ability of trained CNN-ELM-BA using the testing set.
Step5: Repeat Step1 to Step4 5 times.
Output: The five trained CNN-ELM-BA structures and the average statistics.

**FIGURE 7:** Flowchart of CNN-ELM-BA.

**TABLE 5:** Pseudocode of determining the best number of layers to be substituted by ELM.

Input: The dataset and the trained CNN.
Step1: For *n* = 3 to 7, repeat Step2 to Step5.
Step2: Use an ELM structure to substitute the last *n* layers of the CNN.
Step3: Optimize the weights and biases in the ELM using the bat algorithm.
Step4: Evaluate the CNN-ELM-BA generalization ability using the testing set.
Step5: Repeat Step2 to Step4 5 times, and obtain the average detection performance of that *n* value.
Step6: Obtain the best *n*^∗^ based on the comparison of the performance of the CNN-ELM-BA with different values of *n*.
Output: The best *n*^∗^.

The article "Cerebral Microbleed Detection via Convolutional Neural Network and Extreme Learning Machine" was retracted in 2023. Reasons: compromised peer review; unreliable results or conclusions.

## Experiment

Our algorithm was implemented based on MATLAB 2021a. The statistical experiment was carried out on a personal computer with i5 8250U CPU, MX150 GPU, and 16GB memory.

### Dataset

After SNP, we finally obtained a CMB dataset of 13,031 samples with 6,407 CMB and 6,624 non-CMB. In the experiments, 9,000 samples were employed for training, and the rest 4,031 samples, served as the testing set. The settings are listed in Table 6. We can see that the volumes of CMB and non-CMB samples are much the same, which is qualified for training and testing.

**TABLE 6:** Dataset and settings.

Total samples			
13,031			
CMB		Non-CMB	
6,407		6,624	
Training		Testing	
9,000		4,031	
CMB	Non-CMB	CMB	Non-CMB
4,214	4,786	2,193	1,838

### CNN-ELM-BA

The hyperparameters for training CNN-ELM-BA are listed below in Table 7. The mini-batch size is 60, because our training set contains only 9,000 samples. The CNN structure consists of 13 layers which is not a big architecture, so the max epoch is defined as 10. In order to accelerate the convergence, the initial learning rate is set as a large value, 1e-2. The hidden node number is the only hyper-parameter in ELM, which was set as 50, following the convention and empirical experience.

**TABLE 7:** Hyperparameters in our method.

	**Hyperparameter**	**Value**
	MiniBatchSize	60
CNN	MaxEpochs	10
	InitialLearnRate	1e-2
ELM	Number of hidden nodes	50
	Number of population	20
	*i_max*	20
	A_0_	1.6
BA	*R*_0_	1e-3
	*A*	0.9
	*Γ*	0.99
	(*f*_*min*_, *f*_*max*_)	(0,2)

For BA optimization, the population size and max iteration are both 20 in considering the computational efficiency. The max pulse loudness, frequency range, and factors follow the default settings.

### Evaluation Statistics

To carry out evaluation and comparison with state-of-the-art methods, we employed three widely used metrics: sensitivity, specificity, and accuracy. The definitions are as follows:


(14) $$S\,e\,n\,s\,i\,t\,i\,v\,i\,t\,y=\frac{T\,P}{T\,P+F\,P}$$

(15) $$S\,p\,e\,c\,i\,f\,i\,c\,i\,t\,y=\frac{T\,N}{T\,N+F\,N}$$

(16) $$A\,c\,c\,u\,r\,a\,c\,y=\frac{T\,P+T\,N}{T\,P+T\,N+F\,P+F\,N}$$

where *TP* and *TN* represent the numbers of correctly classified CMB and non-CMB cases, respectively, and *FP* and *FN* stand for the numbers of misclassified CMB and non-CMB cases, respectively.

The article "Cerebral Microbleed Detection via Convolutional Neural Network and Extreme Learning Machine" was retracted in 2023. Reasons: compromised peer review; unreliable results or conclusions.

### Results and Discussion

### CNN

We construct the CNN architecture according to the settings in Table 3 and run the CNN training and testing five times to obtain the average performance, shown in Table 8. The CNN training result of one time is given in Figure 8. We can see that the training accuracy soared in epoch 1 and 2, and increased marginally afterward.

**TABLE 8:** Performance of CNN (five runs).

Run	Sensitivity	Specificity	Accuracy
1	89.69%	97.88%	93.43%
2	94.57%	85.75%	90.55%
3	96.26%	70.24%	84.40%
4	97.90%	76.01%	87.92%
5	86.23%	86.89%	86.53%
Average	92.93%	83.35%	88.56%

**FIGURE 8:** Training plot of the CNN. **(A)** Diagram of training accuracy and loss. **(B)** Legend.

The testing confusion matrix on the testing set of five runs is given in Table 9, and we can calculate the overall accuracy is 88.56%, the specificity is 83.35%, and sensitivity is 92.93%.

**TABLE 9:** Confusion matrix of CNN (five runs).

		Predicted label	
		Non-CMB	CMB
Actual label	Non-CMB	7,660	1,530
	CMB	775	10,190

### Weight Visualization in CNN

The explanation of CNN is an important topic in deep learning because CNN models can produce promising classification performance, but it is unknown why they make it. Therefore, we tried to provide an interpretation by visualization of the weights in the first convolutional layer in Figure 9. There are only two kernels in the first convolutional layer. It can be observed that the general patterns for classifying CMB and non-CMB are learned by CNN. This good feature generation ability contributes to the classification of our CMB detection system.

**FIGURE 9:** Weight visualization of first convolutional layer.

### CNN-ELM-BA

We run the CNN-ELM-BA five times and obtain the average performance. The results of the five runs are shown in Table 10. The overall classification performance of CNN-ELM-BA on the testing set is illustrated below in Table 11. The accuracy is 95.25%, specificity is 96.10%, and sensitivity is 94.53%, which is better than CNN. The fully connected layers in the CNN were used for classification, so we replace them with the ELM structure. Then, the ELM was further optimized by bat algorithm. The ELM was a classical structure, so the overfitting can be avoided when training the ELM with our CMB dataset. Together, the classification performance was improved.

**TABLE 10:** Results of CNN-ELM-BA (five runs).

Run	Sensitivity	Specificity	Accuracy
1	94.67%	95.70%	95.14%
2	95.26%	96.84%	95.98%
3	92.93%	96.63%	94.62%
4	95.03%	94.94%	94.99%
5	94.76%	96.41%	95.51%
Average	94.53%	96.10%	95.25%

**TABLE 11:** Confusion matrix of CNN-ELM-BA (five runs).

		Predicted label	
		Non-CMB	CMB
Actual label	Non-CMB	8,832	358
	CMB	600	10,365

Figure 10 gives some misclassified samples. It can be seen that these samples are in complex conditions, so our method made the wrong predictions. Our future research will focus on these hard samples.

The article "Cerebral Microbleed Detection via Convolutional Neural Network and Extreme Learning Machine" was retracted in 2023. Reasons: compromised peer review; unreliable results or conclusions.

**FIGURE 10:** Misclassified samples. **(A)** CMB. **(B)** Non-CMB.

### Optimal-Replacing Layers

In order to find the best-replacing layers, we carried out an experiment and recorded the average statistics of 5 runs, shown in Table 12 and Figure 11. The feature denotes the input to the ELM. It is obvious that the accuracy firstly increased with the number of replaced layers and decreased after reaching the peak value at five replaced layers. The former layers in CNN are related to feature extraction, which is significant for classification. The feature dimension in these layers is high, which requires much memory and increases the computational complexity. So those layers should not be replaced by ELM. The structure after the last fifth layer in CNN serves as the classifier, so the feature dimension remains fixed. Therefore, we chose to replace the last five layers with the ELM as it outperformed other alternatives.

**TABLE 12:** Classification performance of our method using different replaced layers (5 Runs).

Layers replaced by ELM	Feature dimension	Accuracy
3	**32**	93.87%
4	**32**	94.45%
**5**	**32**	**95.25%**
6	3,698	88.73%
7	3,872	86.18%

*Bold means the best.*

**FIGURE 11:** Performance of our method using different replaced layers.

### Comparison With State-of-the-Art Approaches

We compared the proposed CMB detection method (CNN-ELM-BA) with other state-of-the-art approaches, including DNN (Hou and Chen, 2016), LReLU (Chen, 2016), and SAR-DNN (Zhang et al., 2017b). The classification performance comparison is given in Table 13 and Figure 12. The datasets in the five listed approaches are from the same source.

**TABLE 13:** Comparison of classification performance for CMB detection.

Methods	Sen	Spe	Acc
DNN (Hou and Chen, 2016)	93.40%	93.05%	93.23%
LReLU (Chen, 2016)	93.05%	93.06%	93.06%
SAR-DNN (Zhang et al., 2017b)	**95.13%**	93.33%	94.23%
CNN (ours)	92.93%	83.35%	88.56%
CNN-ELM-BA (ours)	94.53%	**96.10%**	**95.25%**

*Bold values denote the best values in each column.*

**FIGURE 12:** Performance comparison with state-of-the-art methods.

All the approaches achieved over 90% accuracy except CNN, which was 88.56%. SAR-DNN yielded the best sensitivity of 95.13%, and the sensitivity of CNN-ELM-BA was marginally worse. For specificity and overall accuracy, CNN-ELM-BA was higher than other algorithms. Hence, our CNN-ELM-BA is an accurate and effective tool for detecting CMB.

The article "Cerebral Microbleed Detection via Convolutional Neural Network and Extreme Learning Machine" was retracted in 2023. Reasons: compromised peer review; unreliable results or conclusions.

## Conclusion

In this paper, we put forward an automated cerebral microbleed detection approach, combined CNN, ELM, and BA. The CNN was trained to extract features from images. We disregarded the fully connected layers of CNN and utilized the ELM for classification. The weights and biases in ELM were optimized by BA. To decide the best number of layers to be replaced by ELM, a searching method was proposed. Our method can be regarded as a general image classification framework, which can be transferred to solve other computer vision tasks. The proposed algorithm yielded an overall accuracy of 95.25%, which was better than three state-of-the-art approaches based on hold-out validation.

However, there are some problems unsolved. First of all, the interpretation of the parameters in the networks is hard, so that we don’t know how or why the prediction is made. Our method can only provide diagnosis results but cannot give an explanation. Moreover, our approach merely solved a binary classification problem, but the multi-class classification is unsolved.

In the future, we shall employ more complex CNN models for feature extraction and improve the performance of ELM with better parameter optimization. We will also try to transfer our method to detect other brain abnormalities like multiple sclerosis and Alzheimer’s disease.

## Data Availability Statement

The original contributions presented in the study are included in the article/supplementary material, further inquiries can be directed to the corresponding author/s.

## Author Contributions

SiL: conceptualization, software, formal analysis, data curation, and writing—original draft. ShL: validation, formal analysis, resources, writing—original draft, visualization, and supervision. S-HW: methodology, investigation, writing—review and editing, and funding acquisition. Y-DZ: methodology, validation, investigation, resources, writing—review and editing, supervision, project administration, and funding acquisition. All authors contributed to the article and approved the submitted version.

## Conflict of Interest

The authors declare that the research was conducted in the absence of any commercial or financial relationships that could be construed as a potential conflict of interest. The handling editor is currently co-organizing a Research Topic with two of the authors, ShL and Y-DZ, and confirms the absence of any other collaboration.

## Publisher’s Note

All claims expressed in this article are solely those of the authors and do not necessarily represent those of their affiliated organizations, or those of the publisher, the editors and the reviewers. Any product that may be evaluated in this article, or claim that may be made by its manufacturer, is not guaranteed or endorsed by the publisher.

The article "Cerebral Microbleed Detection via Convolutional Neural Network and Extreme Learning Machine" was retracted in 2023. Reasons: compromised peer review; unreliable results or conclusions.

## References

[B1] BarnesS. R. HaackeE. M. AyazM. BoikovA. S. KirschW. KidoD. (2011). Semiautomated detection of cerebral microbleeds in magnetic resonance images. *Magn. Reson. Imaging* 29 844–852. 10.1016/j.mri.2011.02.028 21571479 PMC3118856

[B2] BianW. HessC. P. ChangS. M. NelsonS. J. LupoJ. M. (2013). Computer-aided detection of radiation-induced cerebral microbleeds on susceptibility-weighted MR images. *Neuroimage Clin.* 2 282–290. 10.1016/j.nicl.2013.01.012 24179783 PMC3777794

[B3] ChenY. (2016). Voxelwise detection of cerebral microbleed in CADASIL patients by leaky rectified linear unit and early stopping: a class-imbalanced susceptibility-weighted imaging data study. *Multimedia Tools Applic.* 77:9.

[B4] ChenY. ChenX.-Q. (2016). Sensorineural hearing loss detection via discrete wavelet transform and principal component analysis combined with generalized eigenvalue proximal support vector machine and Tikhonov regularization. *Multimedia Tools Applic.* 77 3775–3793. 10.1007/s11042-016-4087-6

[B5] ChenY. Villanueva-MeyerJ. E. MorrisonM. A. LupoJ. M. (2018). Toward automatic detection of radiation-induced cerebral microbleeds using a 3D deep residual network. *J. Digit. Imaging* 32 766–772. 10.1007/s10278-018-0146-z 30511280 PMC6737152

[B6] ChesebroA. G. AmaranteE. LaoP. J. MeierI. B. MayeuxR. BrickmanA. M. (2021). Automated detection of cerebral microbleeds on T2^∗^-weighted MRI. *Sci. Rep.* 11:4004.10.1038/s41598-021-83607-0PMC788986133597663

[B7] FazlollahiA. MeriaudeauF. GiancardoL. VillemagneV. L. RoweC. C. YatesP. (2015). Computer-aided detection of cerebral microbleeds in susceptibility-weighted imaging. *Comput. Med. Imaging Graph.* 46 269–276. 10.1016/j.compmedimag.2015.10.001 26560677

[B8] GolestanehP. ZekriM. SheikholeslamF. (2018). Fuzzy wavelet extreme learning machine. *Fuzzy Sets Syst.* 342 90–108. 10.1016/j.fss.2017.12.006

[B9] Guang-BinH. Qin-YuZ. Chee-KheongS. (2006). Extreme learning machine: theory and applications. *Neurocomputing* 70 489–501. 10.1016/j.neucom.2005.12.126

[B10] HeK. ZhangX. RenS. SunJ. (2016). “Deep residual learning for image recognition,” in *Proceedings of the IEEE Conference on Computer Vision and Pattern Recognition (CVPR)*, (Iowa City, IA: IEEE), 770–778.

[B11] HongJ. (2018a). Classification of cerebral microbleeds based on fully-optimized convolutional neural network. *Multim. Tools Appl.* 79 15151–15169. 10.1007/s11042-018-6862-z

[B12] HongJ. (2018b). Sensorineural hearing loss identification via nine-layer convolutional neural network with batch normalization and dropout. *Multim. Tools Appl.* 79 15135–15150. 10.1007/s11042-018-6798-3

The article "Cerebral Microbleed Detection via Convolutional Neural Network and Extreme Learning Machine" was retracted in 2023. Reasons: compromised peer review; unreliable results or conclusions.

[B13] HongJ. (2019). Detecting cerebral microbleeds with transfer learning. *Mach. Vis. Appl.* 30 1123–1133. 10.1007/s00138-019-01029-5

[B14] HongJ. HongC. WangS. H. LiuJ. (2019). Improvement of cerebral microbleeds detection based on discriminative feature learning. *Fund. Inform.* 168 231–248. 10.3233/fi-2019-1830

[B15] HouX.-X. ChenH. (2016). “Sparse Autoencoder based deep neural network for voxelwise detection of cerebral microbleed,” in *Proceedings of the 22nd International Conference on Parallel and Distributed Systems*, (Wuhan: IEEE).

[B16] HuangG. HuangG. B. SongS. YouK. (2015). Trends in extreme learning machines: a review. *Neural Netw.* 61 32–48. 10.1016/j.neunet.2014.10.001 25462632

[B17] HuangG. LiuZ. van der MaatenL. WeinbergerK. Q. (2016). “Densely connected convolutional networks,” in *Proceedings of the IEEE Conference on Computer Vision and Pattern Recognition (CVPR)*, (Iowa City, IA: IEEE).

[B18] HuangG.-B. ChenL. SiewC.-K. (2006a). Universal approximation using incremental constructive feedforward networks with random hidden nodes. *IEEE Trans. Neural Netw.* 17 879–892. 10.1109/tnn.2006.875977 16856652

[B19] HuangG.-B. ZhuQ.-Y. SiewC.-K. (2006b). “Extreme learning machine: a new learning scheme of feedforward neural networks,” in *Proceedings of the International Joint Conference on Neural Networks (IJCNN2004)*, (Iowa City, IA: IEEE), 985–990.

[B20] HuangJ. YuZ. L. GuZ. (2018). A clustering method based on extreme learning machine. *Neurocomputing* 277 108–119.

[B21] JiangY. Y. (2017). Cerebral micro-bleed detection based on the convolution neural network with rank based average pooling. *IEEE Access* 5 16576–16583.

[B22] KaaouanaT. BertrandA. OuamerF. Law-YeB. PyatigorskayaN. BouyahiaA. (2016). Improved cerebral microbleeds detection using their magnetic signature on T2^∗^-phase-contrast: a comparison study in a clinical setting. *NeuroImage Clin.* 15 274–283. 10.1016/j.nicl.2016.08.005 28560152 PMC5435598

[B23] KrizhevskyA. SutskeverI. HintonG. (2012). “Imagenet classification with deep convolutional neural networks,” in *Proceedings of the International Conference on Neural Information Processing Systems*, (Iowa City, IA: IEEE), 1097–1105.

[B24] KuijfH. J. de BresserJ. GeerlingsM. I. ConijnM. M. ViergeverM. A. BiesselsG. J. (2012). Efficient detection of cerebral microbleeds on 7.0 T MR images using the radial symmetry transform. *Neuroimage* 59 2266–2273. 10.1016/j.neuroimage.2011.09.061 21985903

[B25] LiM.-B. HuangG. B. SaratchandranP. SundararajanN. (2005). Fully complex extreme learning machine. *Neurocomputing* 68 306–314. 10.1016/j.neucom.2005.03.002

The article "Cerebral Microbleed Detection via Convolutional Neural Network and Extreme Learning Machine" was retracted in 2023. Reasons: compromised peer review; unreliable results or conclusions.

[B26] LiW. (2019). A gingivitis identification method based on contrast-limited adaptive histogram equalization, gray-level co-occurrence matrix, and extreme learning machine. *Int. J. Imaging Syst. Technol.* 29 77–82. 10.1002/ima.22298

[B27] LiY. XieW. LiH. (2017). Hyperspectral image reconstruction by deep convolutional neural network for classification. *Pattern Recogn.* 63 371–383. 10.1016/j.patcog.2016.10.019

[B28] LiuA. J. (2017). Tea category identification using computer vision and generalized eigenvalue proximal SVM. *Fund. Inform.* 151 325–339. 10.3233/fi-2017-1495

[B29] LiuH. RashidT. HabesM. (2020). “Cerebral microbleed detection via fourier descriptor with dual domain distribution modeling,” in *Proceedings of the 2020 IEEE 17th International Symposium on Biomedical Imaging Workshops (ISBI Workshops)*, (Iowa City, IA: IEEE), 1–4.

[B30] LiuT. KasuL. L. C. HuangG. B. LinZ. (2018). Extreme learning machine for joint embedding and clustering. *Neurocomputing* 277 78–88. 10.1016/j.neucom.2017.01.115

[B31] NogueiraK. PenattiO. A. B. dos SantosJ. A. (2017). Towards better exploiting convolutional neural networks for remote sensing scene classification. *Pattern Recogn.* 61 539–556. 10.1016/j.patcog.2016.07.001

[B32] OurselinS. JoyA. MagrathE. ButmanJ. A. PhamD. L. (2015). Cerebral microbleed segmentation from susceptibility weighted images. *Med. Imaging* 9413:94131E.

[B33] PanH. ZhangC. TianY. (2014). RGB-D image-based detection of stairs, pedestrian crosswalks and traffic signs. *J. Vis. Commun. Image Represent.* 25 263–272. 10.1016/j.jvcir.2013.11.005

[B34] SimonyanK. ZissermanA. (2015). “Very deep convolutional networks for large-scale image recognition,” in *Proceedings of the International Conference on Learning Representations*, (Iowa City, IA: IEEE).

[B35] SuiY. X. (2018). Classification of Alzheimer’s disease based on eight-layer convolutional neural network with leaky rectified linear unit and max pooling. *J. Med. Syst.* 42:85.10.1007/s10916-018-0932-729577169

[B36] SunJ. XiaoZ. XieY. (2017). Automatic multi-fault recognition in TFDS based on convolutional neural network. *Neurocomputing* 222 127–136.

[B37] WangS. DuS. AtanganaA. AijunL. ZeyuanL. (2018). Application of stationary wavelet entropy in pathological brain detection. *Multim. Tools Appl.* 77 3701–3714. 10.1007/s11042-016-3401-7

[B38] XiaM. (2019). Density-based semi-supervised online sequential extreme learning machine. *Neural Comput. Appl.* 32 7747–7758. 10.1007/s00521-019-04066-3

[B39] YangR. XuS. FengL. (2018). An ensemble extreme learning machine for data stream classification. *Algorithms* 11 107–123. 10.3390/a11070107

[B40] YangX.-S. (2010). A new metaheuristic bat-inspired algorithm. *Nat. Inspired Cooperat. Strateg. Optim.* 284 65–74. 10.1007/978-3-642-12538-6_6

The article "Cerebral Microbleed Detection via Convolutional Neural Network and Extreme Learning Machine" was retracted in 2023. Reasons: compromised peer review; unreliable results or conclusions.

[B41] YuX. WangS.-H. (2019). Abnormality diagnosis in mammograms by transfer learning based on ResNet18. *Fund. Inform.* 168 219–230. 10.3233/fi-2019-1829

[B42] ZhanT. M. ChenY. (2016). Multiple sclerosis detection based on biorthogonal wavelet transform, rbf kernel principal component analysis, and logistic regression. *IEEE Access* 4 7567–7576. 10.1109/access.2016.2620996

[B43] ZhangY.-D. HouX.-X. YiC. HongC. MingY. YangJ. (2017a). Voxelwise detection of cerebral microbleed in CADASIL patients by leaky rectified linear unit and early stopping. *Multim. Tools Appl.* 77 21825–21845. 10.1007/s11042-017-4383-9

[B44] ZhangY.-D. ZhangY. HouX.-X. ChenH. WangS.-H. (2017b). Seven-layer deep neural network based on sparse autoencoder for voxelwise detection of cerebral microbleed. *Multim. Tools Appl.* 77 10521–10538. 10.1007/s11042-017-4554-8

[B45] ZouW. YaoF. ZhangB. HeC. GuanZ. (2017). Verification and predicting temperature and humidity in a solar greenhouse based on convex bidirectional extreme learning machine algorithm. *Neurocomputing* 249 72–85. 10.1016/j.neucom.2017.03.023

